RETRACTED

# The Role and Clinical Value of Optimized Fetal Main Pulmonary Artery Doppler Parameters in the Diagnosis and Prognosis Monitoring of Neonatal Respiratory Distress Syndrome

**DOI:** 10.1155/2022/1682225

**Published:** 2022-08-08

**Authors:** Qing Li, Lin Xu, Liang Zhang

**Affiliations:** ^1^Department of Obstetrics, The Maternal and Child Health Hospital of Hunan Province, Changsha 410008, China; ^2^Department of Pediatrics, The Second People's Hospital of Hunan Province, Changsha 410000, China; ^3^Department of Gynecology, The Maternal and Child Health Hospital of Hunan Province, Changsha 410008, China

## Abstract

**Objective:**

A retrospective study was conducted to explore the role and clinical value of optimized fetal main pulmonary artery Doppler parameters in the diagnosis and prognosis monitoring of neonatal respiratory distress syndrome (NRDS).

**Methods:**

Pregnant women admitted to our hospital for delivery from March 2019 to June 2021 were included in the study. There were 372 singleton pregnant women who voluntarily underwent ultrasound and Doppler examinations with informed consent for the study. The AT/ET ratio of the middle segment of the main pulmonary artery, the middle part of the left (or right) pulmonary artery, and the proximal segment of the intrapulmonary artery was measured by ultrasonic Doppler. According to the outcome of the newborn, it was divided into NRDS group (*n* =90) and non-NRDS group (*n* =282) to compare the differences of fetal AT/ET ratio at three Doppler sampling locations and the differences of fetal AT/ET ratio in different gestational weeks. Using Pearson's correlation analysis, the correlation among the Doppler parameters of fetal main pulmonary artery, the ratio of AT and AT/ET, gestational weeks, and the efficiency of prenatal prediction of NRDS was evaluated by receiver-operating characteristic (ROC). In addition, the diagnostic efficiency of fetal main pulmonary artery Doppler parameter AT/ET ratio and amniotic fluid method for prenatal prediction of NRDS was compared.

**Results:**

Compared with the non-NRDS group, the gestational age, gestational age at delivery, and birth weight in the NRDS group were significantly lower than those in the non-NRDS group. The 1 min Apgar score of newborns was less than 7, and the proportion of newborns transferred to NICU was significantly higher than that in the control group. Compared with non-NRDS group, AT was significantly shortened, AT/ET ratio was significantly decreased, and ET was significantly prolonged in NRDS group. The fetal aortic blood flow parameters AT, ET, and AT/ET ratio in different gestational weeks were significantly different among the three groups. The AT/ET ratio in the middle segment of the aorta in NRDS group was lower than that in non-NRDS group. The ratio of AT/ET was still correlated with the occurrence of postpartum NRDS. The AUC value of NRDS predicted by AT/ET ratio was 0.984. In the combined determination of amniotic fluid Lh and S ratio and PG, the diagnostic accuracy of prenatal prediction of neonatal respiratory distress syndrome was 100.005%, 98.43%, and 95.56%, respectively. The accuracy of fetal aortic AT/ET ratio in prenatal prediction of neonatal respiratory distress syndrome was 100.005%, 95.28%, and 95.57%, respectively. The order of Kappa coefficient from high to low was amniotic fluid PG/L/S ratio, fetal main pulmonary artery blood flow parameter AT/ET ratio, amniotic fluid L/S ratio, OD650, amniotic fluid PG, and foam test.

RETRACTED

**Conclusion:**

Fetal main pulmonary artery Doppler AT/ET ratio may be a very potential parameter for prenatal noninvasive prediction of NRDS. The fetal main pulmonary artery Doppler flow spectrum may be a very potential alternative to amniocentesis to evaluate FLM.

## 1. Introduction

Neonatal respiratory distress syndrome (NRDS) is a respiratory disease that seriously threatens the lives of newborns, especially premature infants [1]. The clinical manifestations are dyspnea, respiratory moan, inspiratory triple indentation sign, and cyanosis, which can easily lead to hyperventilation, hypoxemia, and respiratory acidosis. If it cannot be controlled in time within 2 days after the onset of the disease, respiratory failure can be caused even leading to death [1, 2]. The occurrence of this disease is related to the mode of delivery, maternal age, multiple births, prenatal corticosteroid use, maternal diabetes, intrauterine infection, and other factors [2]. The disease often occurs in premature infants, the younger the gestational age, the higher the incidence [3, 4]. In recent years, the probability of newborns suffering from NRDS has a remarkable increasing trend [5–7]. The disease is a common disease in neonatal intensive care unit, which is one of the main causes of death of newborns, especially premature infants [8, 9]. Therefore, early diagnosis and taking appropriate measures as soon as possible are particularly important to reduce the mortality with NRDS.

Up to now, prenatal assessment of fetal lung maturity to predict the risk of NRDS is very important to prevent the occurrence of NRDS [10]. At present, the clinical evaluation of fetal lung maturity (FLM) mainly depends on amniocentesis for amniotic fluid analysis, including determination of amniotic fluid lecithin/sphingomyelin ratio, detection of phosphatidylglycerol, and the optical density value (OD650) of 650 nm measured by foam test and spectrophotometer. Among them, the determination of liquid chromatograph mass spectrometry (LCMS) and prostaglandins (PG) is the “gold standard” for judging FLM [11]. However, using thin layer chromatography (TLC) to determine L/S ratio and PG, the test process is tedious and time-consuming. The quality control of the test process is not easy and the interpretation of the results is subjective, resulting in large differences in sensitivity and specificity among laboratories [12]. Although amniotic fluid foam test and OD650 measurement have the advantages of simplicity and rapidness, compared with L/S and PG measurements, however, the positive predictive value for predicting fetal lung immaturity is only 13% to 29.5%. It is remarkably lower than L/S and PG (23%-53%). Therefore, it still cannot replace the determination of L/S and PG. In addition, the above methods for evaluating FLM require invasive amniocentesis.

RETRACTED

In order to reduce the incidence of NRDS, glucocorticoid is routinely given to pregnant women at high risk of NRDS to promote fetal lung maturation. However, corticosteroids are not completely without side effects. Leung-Pineda et al. concluded that although the FLM test has been reduced in recent years, it is still impossible to abandon the test in the foreseeable future [13]. It can be noticed that there is an urgent need to develop noninvasive prenatal assessment FLM methods to meet clinical needs, make corticosteroid treatment more targeted, and avoid abuse.

Ultrasound was once considered a “restricted area” for the diagnosis of lung diseases. In recent years, many scholars have been devoted to the in-depth study of lung ultrasound examination [13]. Compared with chest X-ray examination, lung ultrasound examination has the advantages of no ionizing radiation exposure, economy, simplicity, repeatability, and bedside dynamic monitoring [14]. In addition, color Doppler can directly display the distribution of blood vessels and accurately evaluate the changes of hemodynamics. Therefore, we can use Doppler to clearly display the fetal pulmonary artery, accurately place the Doppler sampling volume, and obtain the blood flow velocity wave form [15]. At present, some scholars have successfully used Doppler to measure the ratio of fetal pulmonary artery acceleration time to ejection time to predict fetal pulmonary dysplasia. Pulmonary artery acceleration time/ejection time (AT/ET) ratio is currently recognized as a noninvasive method for evaluating pulmonary artery pressure. Some scholars have reported the use of AT/ET ratio to predict the occurrence of NRDS [16, 17]. In addition, Doppler measurement of pulmonary artery in postnatal newborns indicated that the AT/ET ratio in NRDS infants was remarkably lower compared to non-NRDS newborns. However, the results of previous studies were shown the opposite, suggesting that the ratio of AT/ET in NRDS group was remarkably higher than non-NRDS group. Therefore, it is necessary to conduct a large-scale prospective study to explore the feasibility of fetal main pulmonary artery Doppler parameters AT/ET in evaluating FLM. Therefore, a retrospective study was conducted to explore the role and clinical value of optimized fetal main pulmonary artery Doppler parameters in the diagnosis and prognosis monitoring of NRDS.

RETRACTED

## 2. Patients and Methods

### 2.1. General Information

A total of 372 singleton pregnant women who gave birth from March 2019 to June 2021 in our hospital and received ultrasound and Doppler examination voluntarily with informed consent were enrolled as subjects. The AT/ET ratio of the middle segment of the main pulmonary artery, the middle part of the left (or right) pulmonary artery, and the proximal segment of the intrapulmonary artery was measured by ultrasonic Doppler. According to the neonatal outcome, the newborns were assigned into NRDS group (*n* =90) and non-NRDS group (*n* =282). The age of pregnant women in NRDS group was from 18 to 40 years old and the average age was 29.15 ± 5.88 years old. The age of pregnant women in non-NRDS group was from 18 to 44 years old with an average age of 30.68 ± 4.62 years. There exhibited no statistical significance in the general data. This study was permitted by the Medical Ethics Association of our hospital.

Selection criteria: (1) newborns who meet the diagnostic criteria of NRDS; (2) newborns with complete clinical data; (3) pregnant women who sign informed consent forms.

Exclusion criteria: (1) fetuses with congenital or cardiac malformations; (2) pregnant women who had undergone Doppler ultrasound examination more than 72 hours before delivery; (3) pregnant women who refused to participate in this study; (4) non-NRDS pregnant women who delivered within 72 hours after prenatal glucocorticoid treatment; 5) those with incomplete clinical data.

### 2.2. Treatment Methods

The Siemens Acuson 512 color Doppler ultrasound diagnostic instrument was used and the frequency of abdominal probe was 2.5~6 MHz. When the pregnant woman was in the supine position, the fetus was calm (no fetal respiratory and limb movement) and sinus rhythm was measured. All the measurements were done by a special person on the same machine.

Ultrasonic examination method: (1) First, fetal large artery malformations and other severe cardiac malformations were excluded by four-chamber cephalic deflection method. The standard transverse or apical four-chamber view was taken and tilted to the cephalic side to obtain the right ventricular outflow tract view, which was slightly rotated to the heart base short axis view to clearly display the main pulmonary artery (showing pulmonary valve and left and right pulmonary artery bifurcation). The left (or right) pulmonary artery and intrapulmonary artery were enrolled to measure the pulmonary artery located in the proximal area and adjust the probe so that the angle between the sound beam and the measured blood vessel is <20°. The image was enlarged as much as possible and the sampling frame was placed in the middle part of the fetal main pulmonary artery, the middle part of the left (or right) pulmonary artery, and the proximal segment of the intrapulmonary artery, respectively. The size was 3 mm and the maximum velocity curve showed that the flow velocity was 100cm/s. The paper speed (Sweep) was set to 200 mm/s and the minimum measurement interval was 1 ms. The peak systolic velocity and early diastolic notch points were clearly displayed by adjusting the gain. (2) After the typical best bimodal velocity curve of fetal pulmonary artery was obtained, the systolic AT (the time from the beginning of pulmonary artery contraction to the first systolic peak) and ET (the time from the beginning to the end of systole) were measured by manual recording. The AT/ET ratio was calculated and the average value was obtained after 3 times of measurement.

RETRACTED

During the postpartum follow-up, the neonatal Apgar score, birth weight, the rate of transfer to neonatal ward, and the diagnosis of neonatal discharge were recorded. The diagnosis of NRDS was confirmed by neonatal pediatricians according to medical history, clinical symptoms, signs, and chest X-ray examination.

### 2.3. Statistical Analysis

SPSS23.0 software was adopted for statistical analysis. The basic information of pregnant women and newborns was collected. The AT/ET ratio of different Doppler sampling positions of fetuses was compared by independent sample *t*-test. In the bivariate correlation analysis of normal distribution using Pearson's correlation analysis, that draw the subject operating characteristic curve, the area under the curve was calculated to determine its predictive efficiency. The tangent point with the largest Youden index was taken as the best diagnostic threshold to calculate the fetal main pulmonary artery Doppler velocity curve AT/ET ratio to predict the sensitivity and specificity of NRDS. Logistic regression analysis was adopted to correct the influence of gestational age to understand the relationship between Doppler parameters and the occurrence of NRDS. When *P* value was less than 0.05, the difference was considered to be statistically remarkable.

RETRACTED

## 3. Results

### 3.1. The Pregnancy Outcome of Pregnant Women

There exhibited no remarkable difference between the NRDS and the non-NRDS group in terms of maternal age and the time interval measured by ultrasound (*P* > 0.05). Compared with non-NRDS group, the gestational age, delivery gestational age, and newborn birth weight in NRDS group were remarkably lower (*P* < 0.05). The rate of conversion to NICU was remarkably higher in newborns with Apgar score < =7 at 1 minute after birth (*P* < 0.05). Compared with the non-NRDS group, the AT in the NRDS group was remarkably shortened, the ratio of AT/ET was remarkably lower, and the ET was remarkably prolonged (*P* < 0.05). All results are indicated in Table 1.

### 3.2. Comparison of Doppler Parameters of Fetal Main Pulmonary Artery in Different Gestational Weeks

We compared the Doppler parameters of fetal main pulmonary artery in different gestational weeks. There were remarkable differences among the three groups of fetal main pulmonary artery Doppler parameters AT, ET, and AT/ET (*P* < 0.05). All the results are indicated in Table 2.

### 3.3. The AT/ET Ratio at Different Doppler Sampling Positions of Fetuses

We compared the AT/ET ratio of different Doppler sampling positions of the fetuses. The AT/ET ratio of the mid-segment main pulmonary artery of the fetus in the NRDS group was lower compared to the non-NRDS group (*P* < 0.05). However, there exhibited no remarkable difference in the AT/ET ratio of fetal left (or right) middle pulmonary artery and proximal pulmonary artery (*P* < 0.05). All results are indicated in Table 3.

### 3.4. The Correlation of Doppler Parameters of Fetal Main Pulmonary Artery

There was a remarkable positive correlation between the Doppler parameters of fetal main pulmonary artery AT and AT/ET and the gestational weeks and the correlation coefficients of Pearson were 0.608 and 0.705, respectively (*P* < 0.001). There was a negative correlation between ET and gestational weeks examined by Doppler ultrasound. The Pearson correlation coefficient was -0.390 (*P* < 0.001). After correcting the influence of gestational age by binary logistic regression analysis, there was still a correlation between AT/ET ratio and the occurrence of postpartum NRDS (*P* < 0.05); however, there exhibited no correlation between AT and ET and postpartum NRDS after correcting the influence of gestational weeks (*P* > 0.05).

### 3.5. The Efficiency of Antepartum Prediction of NRDS by AT/ET Ratio of Doppler Velocity Curve of Fetal Main Pulmonary Artery

ROC curve analysis indicated that the AUC of fetal main pulmonary artery Doppler parameter AT/ET ratio for prenatal prediction of NRDS was 0.984 (95% CI 0.958~1.000, *P* < 0.05). Taking the cut-off point of the largest Youden index as the cut-off value, the AT/ET ratio < =0.2175 was used to predict the occurrence of NRDS. The sensitivity and specificity were 93.31% and 95.92%. All the results are indicated in Figure 1.

RETRACTED

### 3.6. The Diagnostic Efficacy of AT/ET Ratio of Fetal Main Pulmonary Artery Doppler Parameters and Amniotic Fluid Method in Prenatal Prediction of NRDS

The sensitivity, specificity, and accuracy of amniotic fluid foam test for prenatal prediction of NRDS were 100%, 52.36%, and 55.87%. The diagnostic efficacy of OD650 in prenatal prediction of NRDS was 80.00%, 88.87%, and 88.36%, respectively. The diagnostic efficacy of amniotic fluid PG in prenatal prediction of NRDS was 100.00%, 77.79%, and 79.43%, respectively. The diagnostic efficacy of amniotic fluid L/S ratio in prenatal prediction of NRDS was 100.00%, 93.66%, and 94.17%, respectively. In the combined determination of amniotic fluid L/S ratio and PG, the diagnostic efficacy of prenatal prediction NRDS was 100.00%, 98.43%, and 98.56%. The diagnostic efficacy of AT/ET ratio of fetal main pulmonary artery in prenatal prediction of NRDS was 100.00%, 95.28%, and 95.57%, respectively. All the results are indicated in Table 4.

### 3.7. Consistency and Differences of Various Methods for Evaluating FLM

We analyzed the consistency and difference of various methods for evaluating FLM. Compared with the actual situation of postnatal clinical diagnosis of NRDS, the consistency and difference of various methods for evaluating FLM, except foam test and amniotic fluid PG test, compared with the actual occurrence of postnatal NRDS, McNemar's test was not statistically remarkable (*P* > 0.05). The Kappa coefficients from high to low were shown as “Joint determination of amniotic fluid PG and L/S ratio,” fetal main pulmonary artery Doppler parameter AT/ET ratio, amniotic fluid L/S ratio, OD650, amniotic fluid PG, and foam test. With the comparison of fetal main pulmonary artery Doppler parameter AT/ET ratio and “combined determination of amniotic fluid PG and L/S ratio” to judge FLM, the two methods were moderately consistent. All the results are indicated in Table 5.

## 4. Discussion

Neonatal respiratory distress syndrome (NRDS) mainly occurs in premature infants [17]. The main causes of NRDS are lack of alveolar surfactant and immature alveolar structure. In recent years, the use of pre-corticosteroids has reduced the incidence of NRDS, but the mortality rate of NRDS remains high, which is still the most important cause of premature infant death [18]. It is very important for clinical diagnosis and treatment to accurately judge the fetal lung maturity of premature infants with gestation of 28 weeks but less than 37 weeks. The traditional detection methods of fetal lung maturity include amniotic fluid oscillation test, amniotic fluid absorbance at 650 nm (A650), amniotic fluid lecithin/sphingomyelin ratio, and phosphatidylglycerol detection [19]. These methods are of high value in the diagnosis of fetal lung maturity, but all of them need amniocentesis and the amniotic fluid extracted cannot be examined in batches [20]. In the meantime, the results of other methods were easily contaminated by meconium and blood; however, the examination of phosphatidylglycerol and lecithin/sphingomyelin ratio was time-consuming, complex, subjective, and lack of quality control [21]. Therefore, the application of traditional fetal lung maturity evaluation method in clinical work is limited.

RETRACTED

For a long time, the clinical diagnosis, curative effect evaluation, and follow-up observation of NRDS are mainly based on the clinical manifestation, blood gas analysis index, and chest X-ray examination [22]. As the main imaging examination method of NRDS, chest X-ray has the advantages of simple operation and convenient use, but it lacks specificity in the early stage. In addition, it is easy for clinicians to have errors in judging the condition [23]. Moreover, X-ray examination has ionizing radiation and newborns are particularly sensitive to it. In order to understand the recovery of the lungs, chest X-ray examination is often needed, which will inevitably lead to high ionizing radiation damage due to many times of X-ray examination [23, 24]. Therefore, there is an urgent need for efficient, convenient, and safe examination methods to study the pulmonary condition of NRDS infants [24].

With the continuous progress of ultrasound diagnosis technology, the artifact of ultrasound in the lung can be adopted to reflect and infer the pathological changes of the lung [25]. It makes it possible to use lung ultrasound as the main means of diagnosing lung diseases in a clinic. At present, lung ultrasound has gradually become research hotspot [26]. The relevant literature has pointed out that the sensitivity and accuracy of lung ultrasound in the diagnosis of pneumothorax are 96.2% and 99.5%, respectively, while the sensitivity and accuracy of chest X-ray diagnosis are 73.1% and 96.5%, respectively. The results showed that the sensitivity of chest X-ray in the diagnosis of pneumothorax is relatively poor [27]. Aafreen S et al. evaluated the diagnostic accuracy of bedside lung ultrasound and chest X-ray in patients with suspected pneumonia through prospective clinical studies [28]. The results indicated that the sensitivity and specificity of bedside chest X-ray in the diagnosis of pneumonia were 67% and 85%, respectively, while the sensitivity and specificity of lung ultrasound were 98% and 95%, respectively. In addition, lung ultrasound also has high value in the diagnosis of a series of lung diseases such as atelectasis, pulmonary edema, acute lung injury, and acute respiratory distress syndrome [29]. At the International Federation of Lung Ultrasound held in 2012, more than 30 medical experts reached a consensus on ultrasonic diagnosis of lung diseases. That showed on the basis of evidence-based medicine for related research, it fully affirmed the value of ultrasound in the diagnosis of lung diseases and strongly promoted the further development of lung ultrasound diagnosis technology [30]. In recent years, pulmonary ultrasound technology has been widely used in a clinic, and it is often used in critical medicine, emergency medicine, respiratory medicine, and other fields, and has achieved good results.

RETRACTED

### 4.1. The Difference of the Results of Color Doppler Ultrasonography among Different Fetuses

Color Doppler flow imaging can directly display the vascular distribution of fetal lung. Due to the high fetal pulmonary artery pressure, the Doppler velocity curve indicated a typical “bimodal”: rapid acceleration reached the first systolic peak velocity in the early systolic period and then decreased due to ventricular contraction, while the second peak appeared in the middle and late systolic period. However, the acceleration is slow and the flow velocity is lower than the first peak velocity. At present, some studies have applied AT/ET ratio to prenatal prediction of pulmonary dysplasia. Luo J H et al. measured fetal main pulmonary artery hemodynamic parameters, including AT/ET ratio, main pulmonary artery plasticity index, and resistance index, before detecting amniotic fluid lecithin/sphingomyelin ratio in 29 singleton pregnant women with indications to evaluate fetal lung maturity. The results indicated that AT/ET ratio and lecithin/sphingomyelin ratio were correlated; there was no correlation between other parameters and lecithin/sphingomyelin ratio. In addition, Spillane N T et al. measured the AT/ET ratio of left (right) pulmonary artery in 163 cases of normal pregnancy and 17 cases of pulmonary dysplasia caused by pulmonary cystadenoma and diaphragmatic hernia. The AT/ET ratio in pulmonary dysplasia group was remarkably lower compared to normal group (0.15 ± 0.02 vs 0.17 ± 0.02); however, as long as the AT/ET ratio of one pulmonary artery was in the normal range, the fetus could survive after birth. The results of these two studies suggested that the AT/ET ratio may have a certain application value in the evaluation of lung maturity. However, the Doppler measurement position is different; the middle left (or right) pulmonary artery and the proximal intrapulmonary artery were measured in 372 premature singletons in order to explore the effect of pulmonary artery Doppler measurement position on the prenatal prediction of NRDS efficiency of AT/ET ratio. In the meantime, a preliminary study was conducted on the efficiency of AT/ET ratio in prenatal prediction of NRDS in premature infants. The results of this study indicated that there exhibited no remarkable difference in the age of pregnant women and the interval between ultrasonic distance and delivery between NRDS group and non-NRDS group (*P* > 0.05). Compared with non-NRDS group, NRDS group indicated remarkably lower gestational age, delivery gestational age, and neonatal birth weight (*P* < 0.05). The newborns with Apgar score < = 7 at 1 minute after birth and the rate of conversion to NICU were remarkably higher (*P* < 0.05). The AT of NRDS group was remarkably shorter than non-NRDS group, the ratio of AT/ET was remarkably lower, while ET was remarkably longer (*P* < 0.05). Comparing the Doppler parameters of fetal main pulmonary artery in different gestational weeks, there were remarkable differences among the three groups of fetal main pulmonary artery Doppler parameters AT, ET, and AT/ET ratio (*P* < 0.05). The AT/ET ratio of the middle segment of main pulmonary artery in NRDS group was lower compared to non-NRDS group (*P* < 0.05). However, there exhibited no remarkable difference in AT/ET ratio between the left (or right) middle pulmonary artery and proximal pulmonary artery (*P* > 0.05). There exhibited a remarkable positive correlation between the Doppler parameters of fetal main pulmonary artery AT and AT/ET and the gestational weeks. The correlation coefficients of Pearson were 0.608 and 0.705, respectively (*P* < 0.001). There exhibited a negative correlation between ET and gestational weeks examined by Doppler ultrasound, and the correlation coefficient of Pearson was -0.390 (*P* < 0.001). After correcting the influence of gestational age by binary Logistic regression analysis, there was still a correlation between AT/ET ratio and postpartum NRDS (*P* < 0.05). However, there exhibited no correlation between AT and ET and postpartum NRDS after correcting the influence of gestational weeks (*P* > 0.05). It has been recognized that AT/ET ratio of pulmonary artery can be adopted for noninvasive evaluation. There is a strong negative correlation between PAP, AT/ET ratio, and PAP. It is generally believed that AT/ET ratio less than 0.4 can be adopted to diagnose pulmonary hypertension. ROC curve analysis indicated that the AUC of fetal main pulmonary artery Doppler parameter AT/ET ratio for prenatal prediction of NRDS was 0.984 (95% CI 0.958~1.000, *P* < 0.05). Taking the maximum tangent point of the Youden index as the cut-off value, the AT/ET ratio < =0.2175 was used to predict the occurrence of NRDS. The sensitivity and specificity were 93.31% and 95.92%, respectively, which were basically consistent with the conclusions of previous studies.

RETRACTED

### 4.2. Analysis of Diagnostic Efficiency of Color Doppler Ultrasound

The efficiency of commonly FLM method is summarized in the ACOG Practice Guide. In addition, it is found that the negative predictive values for predicting fetal lung maturation are very high (95%-100%), but the positive predictive values for immature prediction are different with the highest L/S ratio and PG. Kulovich et al. found that the sensitivity of detecting PG while measuring L/S ratio was unchanged, but it could improve the specificity of the test. The results of this study were consistent with those reported in the literature, which confirmed that “combining L/S ratio and PG” was the most accurate amniotic fluid analysis method for prenatal prediction of NRDS. However, the test process of amniotic fluid L/S ratio and PG detection based on TLC technology was tedious and time-consuming, and the test process was not easy to quality control, which limited its clinical application. In contrast, although foam test and OD650 determination are less specific in predicting NRDS, they are simple and rapid. K J et al. simultaneously detected the OD650 values of 131 amniotic fluid samples and 108 foam tests, all of which were collected within 48 hours before delivery. The accuracy of predicting NRDS was 95% and 56%, respectively. The results of this study show that the diagnostic efficacy of OD650 in postpartum NRDS is more suitable to be used as a clinical diagnostic index. The consistency of OD650 in diagnosing postpartum NRDS is better than that of foam test. The results showed that the efficiency of prenatal prediction of NRDS by using fetal Doppler main pulmonary artery parameter AT/ET ratio was equivalent to that of the gold standard “combined determination of amniotic fluid L/S ratio and PG “efficiency of FLM detection. There exhibited no statistical difference between the two methods in McNemar's test and the Kappa coefficient was 0.682. Compared with the actual situation of postnatal NRDS, the Kappa coefficient of AT/ET ratio for prenatal prediction of NRDS was as high as 0.748. Our study still has some shortcomings. Firstly, the quality of this study is limited due to the small sample size we included in the study. Secondly, this research is a single-center study and our findings are subject to some degree of bias. Therefore, our results may differ from those of large-scale multicenter studies from other academic institutes. Our research is still clinically significant and further in-depth investigations will be carried out in the future.

RETRACTED

In conclusion, fetal main pulmonary artery Doppler AT/ET ratio may be a very potential parameter for prenatal noninvasive prediction of NRDS. The fetal main pulmonary artery Doppler flow spectrum may be a very potential alternative to amniocentesis to evaluate FLM.

## Figures and Tables

**Figure 1:** Doppler velocity curve of fetal main pulmonary artery AT/ET ratio to predict the ROC curve of NRDS.

**Table 1:** Basic information and pregnancy outcome of pregnant women in two groups.

Grouping	NRDS (*n* =90)	Non-NRDS (*n* =282)	*t*/*χ*2	*P*
Pregnant woman's age (age)	29.15 ± 5.88	30.68 ± 4.62	*1.224*	*>0.05*
Ultrasonic measurement of gestational age (weeks)	29.07 ± 2.03	37.71 ± 2.44	*16.140*	*<0.05*
Gestational week of delivery (week)	29.54 ± 2.07	38.06 ± 2.31	*16.312*	*<0.05*
Interval between ultrasound and delivery (weeks)	0.47 ± 0.43	0.38 ± 0.31	*1.017*	*>0.05*
Birth weight (g)	1347.22 ± 330.61	3206.78 ± 627.45	*9.372*	*<0.05*
1 minute Apgar ≤7 (%)	70 (77.78)	8 (2.84)	*231.227*	*<0.05*
Conversion rate to NICU (%)	90 (100.00)	93 (32.98)	*122.616*	*<0.05*
AT (ms)	37.35 ± 3.84	45.18 ± 3.72	*8.536*	*<0.05*
ET (ms)	191.83 ± 13.69	177.05 ± 8.56	*6.784*	*<0.05*
AE/ET ratio	0.18 ± 0.02	0.26 ± 0.02	*13.268*	*<0.05*

**Table 2:** Comparison of Doppler parameters of fetal main pulmonary artery in different gestational weeks [$\bar{x}\pm s$].

Group	N	AT (ms)	ET (ms)	AE/EY ratio
<34 weeks	196	39.16 ± 4.42^∗∗^^, #^	187.23 ± 12.31^∗∗^^, #^	0.21 ± 0.02^∗∗^^, #^
34 weeks 36+6 weeks	95	42.98 ± 2.71^∗^^, #^	176.13 ± 8.89^∗^	0.26 ± 0.02^∗^
≥37 weeks	81	46.08 ± 3.54^∗^^,^ ^∗∗^	176.32 ± 8.13^∗^	0.24 ± 0.01^∗^^,^ ^∗∗^
*F*		123.436	137.625	198.316
*P*		<0.05	<0.05	<0.05

Note: compared with <34 weeks, ^∗^*P* < 0.05; compared with 34 weeks, 36^+ 6^ weeks,^∗∗^*P* < 0.05; compared with ≥37 weeks, ^#^*P* < 0.05.

**Table 3:** The AT/ET ratio at different Doppler sampling positions between two groups of fetuses [$\bar{x}\pm s$].

Group	*N*	Middle segment of fetal main pulmonary artery	The middle segment of the left (or right) pulmonary artery of the fetus	Proximal segment of fetal intrapulmonary artery
NRDS group	90	0.19 ± 0.01	0.16 ± 0.03	0.14 ± 0.01
Non-NRDS group	282	0.25 ± 0.02	0.17 ± 0.04	0.15 ± 0.04
*t*		18.935	1.183	1.416
*P*		<0.05	>0.05	>0.05

RETRACTED

**Table 4:** AT/ET ratio of fetal main pulmonary artery Doppler parameters and amniotic fluid to evaluate the diagnostic efficacy of FLM.

Evaluate the FLM method	Clinical outcome		Diagnostic performance parameters (%)		
	NRDS	Non-NRDS	Sensitivity	Specificity degree	Accuracy
Foam test			100	52.36	55.87
Immature	90	134			
Mature	0	148			
OD650			80.00	88.87	88.36
<0.150	70	31			
≥0.150	20	251			
Amniotic fluid PG			100	77.79	79.43
Negative	90	63			
Positive	0	219			
Amniotic fluid LBG S ratio			100	93.66	94.17
<2	90	18			
≥ 2 or 3	0	264			
Combination of PG and L/S			100	98.43	98.56
Immature	90	4			
Mature	0	278			
Doppler AE/ET			100	95.28	95.57
≤0.2175	90	13			
>0.2175	0	269			

**Table 5:** Compared with the actual situation of postnatal clinical diagnosis of NRDS, the consistency and differences of various evaluation methods of FLM.

Evaluate the FLM method	McNemar's test (*P* value)	Kappa coefficient	Degree of consistency
Foam test	<0.001	0.142	Weak
OD650	0.075	0.445	Moderate
Amniotic fluid PG	<0.001	0.339	Weak
Amniotic fluid L/S ratio	0.131	0.679	Height
Combination of PG and L/S	1.000	0.901	Extremely strong
Doppler AE/ET ratio of fetal main pulmonary artery	0.262	0.752	Height

## Data Availability

No data were used to support this study.
